The article "Evaluation of DNA Damage, Biomarkers of Oxidative Stress, and Status of Antioxidant Enzymes in Freshwater Fish (Labeo rohita) Exposed to Pyriproxyfen" was published in 2022. Journal: Oxid Med Cell Longev.

# Evaluation of DNA Damage, Biomarkers of Oxidative Stress, and Status of Antioxidant Enzymes in Freshwater Fish (*Labeo rohita*) Exposed to Pyriproxyfen

**DOI:** 10.1155/2022/5859266

**Published:** 2022-06-10

**Authors:** Xuwen Li, Sumaira Naseem, Riaz Hussain, Abdul Ghaffar, Kun Li, Ahrar Khan

**Affiliations:** ^1^Institute of Traditional Chinese Veterinary Medicine, College of Veterinary Medicine, Nanjing Agricultural University, Nanjing 210095, China; ^2^MOE Joint International Research Laboratory of Animal Health and Food Safety, College of Veterinary Medicine, Nanjing Agricultural University, Nanjing 210095, China; ^3^Department of Zoology, The Islamia University of Bahawalpur, 63100, Pakistan; ^4^Department of Pathology, Faculty of Veterinary and Animal Sciences, The Islamia University of Bahawalpur, 63100, Pakistan; ^5^Faculty of Veterinary Science, University of Agriculture, Faisalabad -38040, Pakistan; ^6^Shandong Vocational Animal Science and Veterinary College, Weifang 261061, China

## Abstract

Pyriproxyfen (PPF) mimics a natural hormone in insects and disrupts their growth. It is a well-known synthetic insecticide and aromatic juvenile hormone analog frequently used in agriculture and vegetable crops to control various insect species. At present, scanty information is available about the possible potential threats of PPF in aquatic organisms. Therefore, in this study, different toxico-pathologic endpoints of PPF like DNA damage, biomarkers of oxidative stress, and status of antioxidant enzymes were determined in *Labeo rohita* (freshwater fish). In our study, 60 active, free from any external obvious ailments, same size, age, and body mass were randomly allocated to four glass aquaria (T0-T3) separately containing 100 L water. The fish present in groups T1, T2, and T3 were administered PPF dissolved in water 300, 600, and 900 *μ*g/L for 30 days. Different tissues including the blood and visceral organs were obtained from each fish on days 10, 20, and 30 of the experiment. Results on various morphological and nuclear changes in red blood cells of PPF-exposed *Labeo rohita* fish including pear-shaped erythrocytes, spherocytes, red blood cells with a blebbed nucleus, micronucleus, and nuclear remnants were significantly increased. Our results on genotoxicity (comet assay) recorded significantly (*P* ≤ 0.05) increased DNA damage in various tissues of insecticide-exposed fish. The results on oxidative stress profile (reactive oxygen species and thiobarbituric acid reactive substances) and antioxidant enzymes (reduced glutathione superoxide dismutase, peroxidase, and catalase) in multiple tissues of *Labeo rohita* fish concluded significantly (*P* ≤ 0.05) higher quantity of biomarkers of oxidative stress and lower concentrations of different antioxidant enzymes in treated fish. Hence, the findings of our experimental research determine that PPF could induce adverse toxic impacts on multiple tissues of *Labeo rohita* fish.

The article "Evaluation of DNA Damage, Biomarkers of Oxidative Stress, and Status of Antioxidant Enzymes in Freshwater Fish (Labeo rohita) Exposed to Pyriproxyfen" was published in 2022. Journal: Oxid Med Cell Longev.

## 1. Introduction

Monitoring of potentially hazardous impacts of different environmental pollutants such as insecticides herbicides, pesticides, and industrial effluents has gotten a lot of attention in the recent several decades all over the world [1–3]. Numerous chemicals have been widely used in public health, agriculture, protection of environmental, aquatic ecosystems, and in different industries for the production of various materials causing great threat to encountered species, biodiversity, and food products [4–6].

The majority of pesticides and insecticides are not biodegradable, and they tend to remain in the soil and water bodies for years [7]. Various chemicals from multiple sources directly and quickly enter into the body of several animals through contaminated water and food products, ultimately inducing different disorders in normal physiological status [1, 8, 9]. Pyriproxyfen (PPF) stimulates a natural hormone in insects that disrupts their growth. It is a well-known aromatic juvenile hormone analog for controlling insect species among other insecticides [10]. Studies have revealed that PPF being a registered insecticide is commonly used in agriculture and on citrus fruit to control a variety of insects like jassids, whitefly, aphids, bollworm, and cutworms throughout the world [11]. Studies indicate that PPF can induce death during mosquito control in different nontarget animals including fish living in the aquatic environments [12]. Previously, different concentrations (89.66 ng/L) of PPF in water samples collected from the river have been detected [13]. Furthermore, the different lethal concentrations of PPF (LC 50) have also been investigated in different species of fish like rainbow trout [14], *Labeo rohita* [15], and embryos of zebrafish [16]. Reports highlighted those different insecticides, herbicides, and pesticides commonly used in various fields like agriculture, industries, and public health adversely affect the early developmental stages of different aquatic animals [17–20]. The direct and indirect exposure to various environmental pollutants causes overproduction and release of reactive oxygen species in animals [21] leading to induction of oxidative stress [1] and depletion of antioxidant enzymes, injury to different organelles of cells including lipids, proteins, and damage to DNA biomolecules [21, 22]. Studies have reported that morphological and nuclear changes in red blood cells, genotoxicity, oxidative stress, and biomarkers of antioxidant enzymes assays are reliable and useful tools for the exact and early screening of toxicity of various synthetic chemicals in birds [23, 24] and other aquatic organisms including fish [21, 25].

The article "Evaluation of DNA Damage, Biomarkers of Oxidative Stress, and Status of Antioxidant Enzymes in Freshwater Fish (Labeo rohita) Exposed to Pyriproxyfen" was published in 2022. Journal: Oxid Med Cell Longev.

DNA damage assessment using comet assay is of great importance and is frequently used in aquatic animals [21, 26, 27]. However, to date, no literature is found in previous data regarding the various toxicological events like nuclear and morphological disorders in red blood cells, oxidative stress, genotoxicity, and status of antioxidant biomarkers due to PPF insecticide in *Labeo rohita*. Therefore, the current study was executed to measure the deleterious effects of PPF on different multiple endpoints including nuclear changes in red blood cells, genotoxicity, oxidative stress, and antioxidant enzymes of *Labeo rohita* fish.

## 2. Materials and Methods

### 2.1. Fish Management

The current study was carried out at the labs of the Islamia University of Bahawalpur's departments of zoology (life sciences) and pathology (veterinary sciences). The total quantity of freshwater fish *Labeo rohita* with body mass (130-140 g), size, and age was collected from a commercial fish farm in the Punjab region of Pakistan (District Bahawalnagar). Following the capture of the fish, all samples were packed in oxygen-rich plastic bags and sent to the laboratory. Fish were housed in a glass tank (10″ L 14″ W 12″ H) for ten days as a means of accommodation. 2-3% food was chosen as body weight and supplied to all of the fishes twice a day, early in the morning, and late in the evening. The aquarium medium was cleaned every day since cleanliness was a big component.

### 2.2. Chemicals

Pyriproxyfen was acquired for research purposes from M/S Ali Akbar Enterprises in Pakistan's main market area of Lodhran. Many more compounds were bought from Merck (Germany) and Sigma Aldrich throughout this investigation (USA). Company (Pvt.) Pakistan provided many commercial kits for the assessment of serum biochemical parameters.

### 2.3. Experimental Strategy and Handling

Following adaption, the fish were chosen at random, separated, and assigned into four groups (T0, T1, T2, and T3). Each had a total of 20 species. Each tank held 100 liters of water. The control group (T0) did not receive PPF dose at any stage and served as negative control. The experimental groups T1, T2, and T3 served as positive groups and received PPF 300, 600, and 900 g/L in distilled water for one month, respectively. Daily, all aquariums were cleansed of residual debris and fecal material for the sake of cleanliness. According to the requirements, all findings and observations were data-recorded each day.

The article "Evaluation of DNA Damage, Biomarkers of Oxidative Stress, and Status of Antioxidant Enzymes in Freshwater Fish (Labeo rohita) Exposed to Pyriproxyfen" was published in 2022. Journal: Oxid Med Cell Longev.

### 2.4. Genotoxicity Assessment and Blood Sampling

On days 10, 20, and 30 of the experiment, each fish was subjected to draw blood from caudal vein utilizing a 26-gauge sterile hypodermic needle. Thin smear from each fish was prepared from fresh blood without the use of any anticoagulant medications to evaluate morphological and nuclear alterations in erythrocytes. The blood films were immediately dried, fixed with 100% alcohol, and stained with Giemsa. A computer-assisted examination of 1500 red blood cells from each fish was carried out using a light microscope with an oil immersion lens [28]. Single-cell gel electrophoresis or the comet test technique were used to evaluate DNA damage in diverse organs such as the liver, gills, and kidneys under alkaline circumstances [29]. After dissection, the liver, kidneys, and gills of each fish were removed and immersed separately in a chilled normal saline solution. The tissues (0.2 g) were combined and homogenized in a centrifuge. Every tissue's single cells was separated and put through a comet test [1]. The slides were rinsed in a cold buffer solution after they were produced. After being lysed, the slides were placed in a horizontal electrophoresis tank with a refrigerated electrophoresis solution. At a voltage of 25 volts, electrophoresis was performed for 25-30 minutes [1]. The slides were after electrophoresis (pH 7.5) and then stained with ethidium bromide solution and viewed at a magnification of 400× using a fluorescence microscope. The range of DNA damage (percent DNA) in each sample was estimated after seeing 500 cells on a fish slide.

### 2.5. Tissue Preparation and Biochemical Analyses

Fish were dissected at days 10, 20, and 30 of the experiment for biochemical analysis. The liver, kidneys, brain, and gills were taken from each fish. All of the tissues were soaked in an ice-cold saline solution. Oxidative stress-causing agents such as reactive oxygen species, lipid peroxidation, thiobarbituric acid reactive species, reduced glutathione, total protein contents, and variant antioxidant enzymes such as superoxide dismutase, catalase, and peroxidase were all examined in samples. Homogenate from various visceral organs was separately prepared, and various antioxidant biomarkers include peroxidase, catalase, superoxide dismutase [1, 30], reduced glutathione [30, 31], and reactive oxygen species [32], and thiobarbituric acid reactive substance [1, 33].

### 2.6. Statistical Analysis

Data thus collected were subjected to statistical analysis by applying ANOVA using SPSS statistics (version 20). The group means were compared by post hoc Tukey's test. Data are presented as mean ± SE. The level of significance was considered at *P* ≤ 0.05.

The article "Evaluation of DNA Damage, Biomarkers of Oxidative Stress, and Status of Antioxidant Enzymes in Freshwater Fish (Labeo rohita) Exposed to Pyriproxyfen" was published in 2022. Journal: Oxid Med Cell Longev.

## 3. Results

### 3.1. Gross Pathology

At necropsy, all the visceral organs such the brain, liver, gills, and kidneys of *Labeo rohita* fish were normal in appearance and consistency throughout the trial. The heart of PPF (900 *μ*g/L) treated *Labeo rohita* exhibited hyperemia, edema, and dark black color after day 20 of the experiment. No obvious gross signs of toxicity of PPF on the liver, brain, and kidneys of *Labeo rohita* are treated with 900 *μ*g/L. The gills of PPF-treated *Labeo rohita* (900 *μ*g/L) were moderately hyperemic. Mild gross signs of toxicity of PPF (600 *μ*g/L) on brain and gills of *Labeo rohita* were observed after day 20 of our study.

### 3.2. Morphological and Nuclear Abnormalities in Red Blood Cells

Results on different cellular abnormalities in erythrocyte of PPF-treated *Labeo rohita* fish at various doses including nuclear abnormalities (erythrocytes with the lobed nucleus, erythrocytes with the blabbed nucleus, notched nucleus, erythrocyte with two nuclei, erythrocyte with micronucleus, and erythrocyte with a condensed nucleus) and morphological abnormalities (pear shape erythrocyte, spindle shape erythrocyte, and spherocyte) are recorded in Table 1 and Figures 1–2. The results exhibited a substantial increase in frequencies of erythrocytes with the lobed nucleus, blabbed nucleus, vacuolated nucleus, and notched nucleus in fish exposed to various amounts of PPF at day 20 in group T2 and at day 30 in group T3 of our research. Notably, the frequencies of formation of micronuclei were substantially high in erythrocytes obtained from fish exposed to PPF in groups T2 and T3 throughout the trial (Figure 1). Remarkably, increased frequencies of erythrocytes with bi-nucleus/dividing nucleus in fish kept in group T3 at day 20 while at day 30 in groups T2 and T3 were recorded (Figure 2). Significantly increased abnormalities in morphology of erythrocyte including pear shape, spindle shape, and spherocyte were detected in blood smear prepared from *Labeo rohita* of fish exposed to higher doses of PPF in comparison to untreated control fish.

### 3.3. Oxidative Stress and Antioxidant Responses

#### 3.3.1. Oxidative Stress and Antioxidant Responses in Liver

The result measured on ROS and TBARS from the liver of PPF-treated fish at day 10 in group T3 and in groups T2 and T3 at days 20 and 30 shows a significantly increased quantity of these biomarkers than the liver obtained from normal *Labeo rohita* fish (Table 2). The result measured on the level of SOD from the liver of PPF-treated fish at day 20 in group T3 and in groups T2 and T3 at day 30 shows a significantly (*P* ≤ 0.05) lower quantity than the liver obtained from untreated organisms. The results measured on the concentration CAT from the liver of PPF-treated fish at day 10 in group T3 and in groups T2 and T3 at days 20 and 30 showed a significantly (*P* ≤ 0.05) reduced quantity than the liver of normal fish. The result computed on the concentration POD from the liver of PPF-treated fish showed significantly (*P* ≤ 0.05) reduced quantity throughout the study in comparison to the normal liver of *Labeo rohita* (Table 2).

The article "Evaluation of DNA Damage, Biomarkers of Oxidative Stress, and Status of Antioxidant Enzymes in Freshwater Fish (Labeo rohita) Exposed to Pyriproxyfen" was published in 2022. Journal: Oxid Med Cell Longev.

#### 3.3.2. Oxidative Stress and Antioxidant Responses in Kidneys

Reduced GSH is a name. Therefore, sentence will beincrease, while in reduced GSH decresaed significantly than the kidneys obtained from normal *Labeo rohita* fish (Table 3). The results of SOD, CAT, and POD from the kidneys of PPF-treated fish at day 20 and 30 in group T2 and T3 showed significantly (*P* ≤ 0.05) lower values than the values obtained from the kidneys of untreated (T0) *Labeo rohita* (Table 3).

#### 3.3.3. Oxidative Stress and Antioxidant Responses in Gills

Our results on oxidative stress biomarkers reveal a significantly (*P* ≤ 0.05) higher quantity of ROS and TBARS from gills of PPF-treated fish at day 30 in groups T2 and T3 than the gills of untreated fish (Table 4). The result recorded on the level of GSH from gills of PPF-treated fish at day 30 in group T3 shows significantly lower values than the gills of unexposed fish at all sampling days. The result obtained at day 10 in fish of group T3 while in groups T2 and T3 at day 20 and on the concentration different antioxidant responses including SOD, CAT, and POD from gills of PPF-treated fish shows significantly (*P* ≤ 0.05) reduced quantity than the gills of *Labeo rohita* (Table 4).

#### 3.3.4. Oxidative Stress and Antioxidant Responses in Brain

We observed a significantly (*P* ≤ 0.05) increased quantity of ROS and TBARS from the brain of PPF-treated fish at days 20 and 30 in groups T2 and T3 and showed significantly increased quantity than the brain of untreated fish (Table 5). The result recorded on the level of GSH from the brain of PPF-treated fish at day 20 in group T3 and at day 30 in groups T2 and T3 indicates significantly lower values than the brain of unexposed fish at all sampling days. The result obtained at day 20 in fish of group T3 while in groups T2 and T3 at day 30 on the concentration different antioxidant responses including SOD, CAT, and POD from the brain of PPF treated fish shows significantly (*P* ≤ 0.05) reduced quantity than the brain of normal fish (Table 5).

### 3.4. DNA Damage Assessment by Comet Assay

The results on DNA damage by comet assay (Figure 3) in different visceral organs of *Labeo rohita* fish treated with various concentrations of PPF showed a significantly (*P* ≤ 0.05) increased percentile rate of DNA damage in isolated cells of the liver, kidneys, and gills at day 10 in group T3 while at day 20 and 30 in groups T2 and T3 compared to untreated fish (Table 6).

The article "Evaluation of DNA Damage, Biomarkers of Oxidative Stress, and Status of Antioxidant Enzymes in Freshwater Fish (Labeo rohita) Exposed to Pyriproxyfen" was published in 2022. Journal: Oxid Med Cell Longev.

## 4. Discussion

The pesticide used unwisely can cause many serious environmental dangers and also pollute the groundwater. These chemical residues do not dissolve in soil for a long period of time and remain in underground water [34]. This contamination is dangerous in agricultural land areas and can be a serious hazard for crops particularly in water resources and should be evaluated in agricultural countries like India and Pakistan [3]. One of these pesticides, PPF is a pesticide that works against a wide range of insects [10]. It was first launched in the USA in 1996 as a whitefly repellent for cotton crops. Other crops have also benefited from it. It is also used to keep domestic pets flea-free, as well as to eliminate ants and roaches both indoors and out [11, 35, 36]. Pyriproxyfen is an insect growth regulator and a juvenile hormone analog [37] that affects their growth. It inhibits larvae from maturing into adults, preventing them from reproducing. Pyriproxyfen damages the liver in mice, rats, and dogs at high dosages surpassing 5000 mg/kg body weight [38].

Therefore, prolonged monitoring and evaluation of the potential toxicity of PPF due to low concentrations of long-term exposure are incredibly important in an attempt to lessen its public health risks. In this research when *Labeo rohita* was treated with PPF, different morphological changes were observed including the pear-shaped nucleus, in different cells, and in some cases, bilobed nucleus like in erythrocyte micronucleus was observed like in red blood cells and in white blood cell types. While in the earlier report, the greater strength of nuclear anomalies including nuclear aberrations of erythrocyte, micronucleus, terminal nucleus, extended and swollen nucleus, and karyopyknotic was observed in silver barb (*Barbonymus gonionotus*) [39] treated with various concentrations of the toxicant. Previously, swollen erythrocytes identified as “spherocytes” change in size and shape of cells like elongated cells, cells with tapered ends, numerous spherocytes, erythrocytes showing contraction from one side and with small projections, the disrupted lipid membrane, and increased lipid peroxidation altered shapes of red blood cells in *Ctenopharyngodon idellus* [1, 40] exposed to the toxicant. Moreover, *Channa punctatus* abnormality occurred in red blood cells (acanthocytes with cytoplasmic blebbing and badly disrupted cell membrane) due to depressed adenosine triphosphate under hypoxic conditions [41] at higher concentrations of the toxicant was found. It was noticed that PPF alone had side effects on fish health; however, the combination of PPF with vitamin E and naringenin used had a better effect on fish health towards recovery.

The article "Evaluation of DNA Damage, Biomarkers of Oxidative Stress, and Status of Antioxidant Enzymes in Freshwater Fish (Labeo rohita) Exposed to Pyriproxyfen" was published in 2022. Journal: Oxid Med Cell Longev.

Under normal physiological conditions, cells are capable of counterbalancing the noxious effects of ROS with the antioxidant defense system which consists of free radical scavengers such as SOD, GSH, glutathione peroxidase (GPx), and CAT. When production of free radicals exceeds the body's antioxidant defense system, it results in oxidative stress [42]. It is imposed on cells due to increase in oxidant generation, a decrease in antioxidant protection, and failure in the repair of oxidative damage [43–46] in the form of severe damage to cellular macromolecules such as proteins, lipids, and DNA, resulting in detrimental effects on cells [47–50]. Pesticides are known to induce ROS and cause oxidative stress in fish [11, 51, 52]. The antioxidant enzymes (SOD, CAT, GPx, and GST) prevent oxidative stress, and the actions of these enzymes are routinely used to monitor the risk of pesticides [53]. Glutathione reductase is a suitable biomarker to evaluate the impact of pesticides in aquatic organisms [54].

The activities of hepatic enzymatic antioxidants SOD, CAT, glutathione peroxidase, glutathione S-transferase, and glutathione reductase were previously examined in similar work. Catalase is a key enzyme that plays an essential role in cell defense against oxidative stress [55]. Several investigators noted changes in liver CAT activity in fish exposed to pesticides and thus considered this enzyme a useful marker of chemical-mediated tissue oxidation [56]. Catalase activity is higher in organs with high oxidative potential such as the liver, kidney, and erythrocytes [57]. Several studies have shown changes in liver catalase of fish exposed to pesticides, and catalase has been considered a useful marker of liver changes due to damage by toxic substances [56, 58].

With a high dose of PPF, the values of the ROS increased considerably in liver tissues. The POD enzymes remarkably reduced in liver of fish received high doses of PPF. In the present study, with little bit different results of parameters like ROS, POD, TBARS were observed in the kidney, gills, and brain. Scanty of work available previously as similar work on different chemicals and species like rats [59] was studied previously. The number of liver cells with damaged DNA increased in this research when the dosage of PPF was increased. The concentrations of ROS and TBARS were assessed in the gills, liver, and kidneys of PPF-treated *Labeo rohita* fish in this study. Previously, no data on PPF-induced oxidative stress (ROS and TBARS) in the *Labeo rohita*'s brain, gills, liver, or kidneys could be located in the literature. However, due to the detoxifying systems of exposed animals, exposure to diverse toxicants produces quick and increased formation of ROS. The formation of ROS starts the process of lipid peroxidation, which leads to cellular membrane irregularities and the development of TBARS [1, 33, 60]. As a result, elevated levels of oxidative stress indices in fish exposed to PPF in the current investigation might be related to antioxidant enzyme depletion and misbalancing. Earlier investigations in rare minnow [61] and bigheaded carp [1] found increased levels of oxidative stress parameters owing to toxicants such as lipid peroxidation product, nitric oxide, and ROS.

The article "Evaluation of DNA Damage, Biomarkers of Oxidative Stress, and Status of Antioxidant Enzymes in Freshwater Fish (Labeo rohita) Exposed to Pyriproxyfen" was published in 2022. Journal: Oxid Med Cell Longev.

Furthermore, several investigations have discovered that DNA damage in various tissues of organisms is mostly caused by the formation of free radicals and oxidative stress [29, 41]. Increased levels of ROS and H_2_O_2_ owing to toxicants have also been observed in rats, which is similar to our findings [62]. ROS production is primarily influenced by toxicant concentrations, cellular backgrounds, duration, and exposure time [1]. Pyriproxyfen also causes oxidative stress by lowering antioxidant enzymes (CAT, SOD, glutathione peroxidase, and glutathione reductase) and increasing lipid peroxidation in both target and non-target animals [11, 63, 64].

Pyriproxyfen, a pesticide and its metabolites, also showed oxidative stress damage by inhibiting the activity of CAT and SOD and increasing MDA [65]. In the present study, fish exposed to PPF caused a decrease in SOD activity in the gill tissue which indicates the adaptive response of fish to pesticides. Catalase (CAT), an important antioxidant enzyme, protects the aquatic organisms from oxidative stress. It catalyzes hydrogen peroxide into water and oxygen consequently completing the detoxification process imitated by SOD [66]. The observed decrease in CAT activity in gill tissue of *Catla catla* treated with ACE and TMX indicates overproduction of ROS due to pesticide stress. Furthermore, inhibition of protein synthesis due to pesticide stress may be another possible reason for the inhibition of CAT activity which has also been reported [67].

The amounts of GSH and total proteins in the gills, livers, and kidneys of fish were shown to be lower in this experimental investigation. To present, there is no information on the effects of PPF on the contents of GSH and total proteins in various *Labeo rohita* tissues. The lower values of GSH and total proteins in various tissues of fish in the current study might be due to dysfunctions of tissues and increased utilization of energy (body proteins) to overcome oxidative stress [64, 68–71]. Previously, it is well-established that different toxicants are responsible for the reduction of proteins in different tissues of fish (*Oreochromis spilurus*, *Mystusvittatus*, *Channa punctatus*, and *Labeo rohita*) including gills, kidneys, and livers [41, 72]. However, other than fish species, DNA damage was also observed in other organisms like birds and mammals [72], rats [6], chickens [73], liver cancer cell line [74, 75], and HepG2 cell line [76]. In contrast to the results on comet assay, no significant increase in DNA damage due to toxicant has been observed in fish [77–79]. Moreover, it can be speculated that DNA damage in different tissues of *Labeo rohita* might also be related to genetic abnormalities induced by PPF leading to the activation of abnormal and physiologically nonfunctional proteins responsible for mitochondrion dysfunctioning and breakage of nuclear proteins [80, 81]. Furthermore, DNA damage in multiple organs of the *Labeo rohita* might be linked to genetic abnormalities generated by PPF, which could lead to the activation of aberrant and physiologically nonfunctional proteins that cause mitochondrion dysfunction and nuclear protein breakdown [1, 82, 83].

The article "Evaluation of DNA Damage, Biomarkers of Oxidative Stress, and Status of Antioxidant Enzymes in Freshwater Fish (Labeo rohita) Exposed to Pyriproxyfen" was published in 2022. Journal: Oxid Med Cell Longev.

## 5. Conclusions

From the findings of the current trial, our results indicated that pyriproxyfen induced deleterious effects on red blood cells and different vital organs of *Labeo rohita*. Exposure of specimen to PPF at 600 *μ*g/L and 900 *μ*g/L causes DNA damage in isolated blood lymphocytes, the brain, gills, liver, and kidneys cells. Moreover, PPF with vitamin C causes low oxidative stress and also causes less reduction in antioxidant enzymes in the brain, livers, kidneys, and gills of *Labeo rohita* in a concentration and time-dependent manner.

## Figures and Tables

**Figure 1:** Blood smear of *Labeo rohita* treated with pyriproxyfen (T3: 900 *μ*g/L at 30 days experiment). Upper and lower figures showing (1) bi-nucleus/dividing nucleus, (2) micronucleus, (3) condensed nuclei, (4) notched nuclei, (5) pear-shaped erythrocyte, and (6) macrocyte (immature erythrocytes). Stain: Giemsa. 1000×.

**Figure 2:** Blood smear of *Labeo rohita* treated with pyriproxyfen (T3: 900 *μ*g/L at 30-day experiment). Upper and lower figures showing (1) notched nucleus, (2) macrocyte (immature erythrocytes), (3) pear-shaped erythrocyte, (4) abnormal erythrocytes, (5) spindle-shaped erythrocyte, (6) elliptical erythrocyte, (7) condensed nuclei, (8) macrocyte, (9) micronucleus, (10) microcyte, and (11) bi-nucleus/dividing nucleus. Stain: Giemsa. 1000×.

The article "Evaluation of DNA Damage, Biomarkers of Oxidative Stress, and Status of Antioxidant Enzymes in Freshwater Fish (Labeo rohita) Exposed to Pyriproxyfen" was published in 2022. Journal: Oxid Med Cell Longev.

**Figure 3:** Comet assay showing DNA damage in isolated cells of the liver of fish treated with pyriproxyfen. (a) 600 *μ*g/L (T2) and (b) 900 *μ*g/L (T3) at 30-day experiment. Note the frequency and intensity is increasing with the dose of pyriproxyfen increasing.

**Table 1:** Various morphological and nuclear alterations in erythrocytes of *Labeo rohita* fish exposed to different pyriproxyfen concentrations.

Parameters/days	Groups/treatment			
	T0 (0.0)	T1 (300 *μ*g/L)	T2 (600 *μ*g/L)	T3 (900 *μ*g/L)
Erythrocytes with lobed nucleus (%)				
10	1.39 ± 0.08	1.42 ± 0.06	1.57 ± 0.09	3.43 ± 0.18∗
20	1.40 ± 0.02	1.43 ± 0.04	1.59 ± 0.08	3.45 ± 0.23∗
30	1.41 ± 0.03	1.47 ± 0.04	3.61 ± 0.09∗	4.46 ± 0.18∗
Erythrocytes with blabbed nucleus (%)				
10	1.22 ± 0.17	1.39 ± 0.22	1.54 ± 0.13	2.99 ± 0.12∗
20	1.24 ± 0.15	1.48 ± 0.17	1.57 ± 0.11	3.18 ± 0.09∗
30	1.29 ± 0.14	1.49 ± 0.16	2.64 ± 0.15∗	3.19 ± 0.07∗
Erythrocytes with vacuolated nucleus (%)				
10	2.36 ± 0.04	2.43 ± 0.02	2.63 ± 0.12	2.99 ± 0.06∗
20	2.38 ± 0.02	2.44 ± 0.04	2.65 ± 0.05	3.03 ± 0.09∗
30	2.40 ± 0.03	2.47 ± 0.04	3.69 ± 0.06∗	3.90 ± 0.16∗
Notched nucleus (%)				
10	1.79 ± 0.01	1.86 ± 0.03	2.92 ± 0.08	2.66 ± 0.10∗
20	1.80 ± 0.02	1.89 ± 0.02	1.95 ± 0.09	2.70 ± 0.07∗
30	1.81 ± 0.01	1.90 ± 0.03	2.67 ± 0.12∗	2.81 ± 0.09∗
Binucleate nucleus (%)				
10	1.44 ± 0.18	1.50 ± 0.13	1.64 ± 0.09	1.77 ± 0.05
20	1.48 ± 0.18	1.55 ± 0.05	1.71 ± 0.09	2.89 ± 0.09∗
30	1.49 ± 0.13	1.63 ± 0.07	3.88 ± 0.05∗	3.91 ± 0.08∗
Pear shaped (%)				
10	3.87 ± 0.34	4.04 ± 0.18	4.10 ± 0.14	7.07 ± 0.04∗
20	3.89 ± 0.31	4.19 ± 0.16	6.68 ± 0.32∗	7.16 ± 0.19∗
30	3.66 ± 0.21	4.20 ± 0.43	6.75 ± 0.28∗	7.19 ± 0.08∗
Micronucleus (%)				
10	1.73 ± 0.18	1.83 ± 0.19	2.24 ± 0.08∗	3.92 ± 0.08∗
20	1.74 ± 0.24	1.96 ± 0.09	2.58 ± 0.13∗	4.04 ± 0.05∗
30	1.75 ± 0.21	2.10 ± 0.13	3.13 ± 0.14∗	4.26 ± 0.06∗
Condensed nucleus (%)				
10	2.11 ± 0.57	2.24 ± 0.21	2.53 ± 0.66	3.41 ± 0.12∗
20	2.30 ± 0.33	2.35 ± 0.51	3.82 ± 0.16∗	4.30 ± 0.05∗
30	2.45 ± 0.48	2.47 ± 0.13	4.95 ± 0.69∗	6.25 ± 0.26∗
Spindle shaped erythrocyte (%)				
10	1.83 ± 0.21	2.09 ± 0.15	3.22 ± 0.19∗	4.40 ± 0.26∗
20	1.95 ± 0.19	2.16 ± 0.19	3.35 ± 0.14∗	4.88 ± 0.21∗
30	1.84 ± 0.34	2.23 ± 0.33	3.49 ± 0.17∗	5.12 ± 0.09∗
Spherocytes (%)				
10	1.94 ± 0.03	2.18 ± 0.17	3.46 ± 0.08∗	4.20 ± 0.23∗
20	1.98 ± 0.08	2.21 ± 0.15	3.56 ± 0.09∗	4.45 ± 0.16∗
30	2.01 ± 0.03	2.25 ± 0.09	3.78 ± 0.16∗	4.69 ± 0.31∗

In each row, values (Mean ± SE) bearing asterisks differ significantly (*P* ≤ 0.05) from that of values in untreated (T0 negative control) fish. T1, T2, and T3 are positive control and dose based.

The article "Evaluation of DNA Damage, Biomarkers of Oxidative Stress, and Status of Antioxidant Enzymes in Freshwater Fish (Labeo rohita) Exposed to Pyriproxyfen" was published in 2022. Journal: Oxid Med Cell Longev.

**Table 2:** Oxidative stress indices and antioxidant enzyme levels in liver tissues of *Labeo rohita* exposed to pyriproxyfen.

Parameters/days	Groups/treatment			
	T0 (0.0)	T1 (300 *μ*g/L)	T2 (600 *μ*g/L)	T3 (900 *μ*g/L)
ROS (optical density)				
10	0.36 ± 0.03	0.37 ± 0.02	0.40 ± 0.03	0.84 ± 0.07∗
20	0.37 ± 0.01	0.39 ± 0.01	0.67 ± 0.02∗	0.86 ± 0.05∗
30	0.39 ± 0.04	0.42 ± 0.03	0.75 ± 0.02∗	0.92 ± 0.05∗
TBARS (nmol/TBARS formed/mg protein/min)				
10	37.42 ± 2.93	39.23 ± 1.95	41.07 ± 1.15	54.93 ± 2.74∗
20	38.89 ± 1.94	40.68 ± 2.95	50.44 ± 1.97∗	56.25 ± 3.92∗
30	40.02 ± 3.94	41.95 ± 2.93	51.88 ± 2.34∗	58.83 ± 4.53∗
Reduced GSH (*μ*mol/g tissue)				
10	8.66 ± 1.17	7.65 ± 0.06	6.64 ± 0.13	5.64 ± 0.15∗
20	8.38 ± 1.12	7.44 ± 1.10	6.05 ± 0.02	5.56 ± 0.12∗
30	8.35 ± 1.14	7.38 ± 1.05	5.93 ± 1.15∗	5.48 ± 0.14∗
*Antioxidant enzymes*				
SOD (units/mg protein)				
10	11.65 ± 0.12	10.97 ± 0.12	10.29 ± 0.13	10.27 ± 0.11
20	11.64 ± 0.15	10.32 ± 0.15	9.46 ± 0.15	7.58 ± 0.14∗
30	10.75 ± 0.18	9.68 ± 0.18	7.10 ± 0.18∗	7.04 ± 0.17∗
CAT (units/min)				
10	8.70 ± 0.19	7.52 ± 0.19	7.14 ± 0.19	5.16 ± 0.19∗
20	7.99 ± 0.17	7.35 ± 0.16	5.63 ± 0.16∗	5.03 ± 0.16∗
30	7.95 ± 0.16	7.02 ± 0.16	5.46 ± 0.16∗	4.95 ± 0.16∗
POD (units/*μ*g)				
10	4.08 ± 0.09	3.56 ± 0.09	2.78 ± 0.09∗	2.47 ± 0.08∗
20	4.03 ± 0.08	3.47 ± 0.08	2.63 ± 0.08∗	2.41 ± 0.08∗
30	3.96 ± 0.08	3.39 ± 0.08	2.55 ± 0.08∗	2.38 ± 0.08∗

In each row, values (Mean ± SE) bearing asterisks differ significantly (*P* ≤ 0.05) from that of values in untreated (T0 negative control) fish. T1, T2, and T3 are positive control and dose based.

**Table 3:** Oxidative stress parameters and antioxidant enzyme levels in *Labeo rohita* kidneys tissues subjected to pyriproxyfen dosages.

Parameters/days	Groups/treatment			
	T0 (0.0)	T1 (300 *μ*g/L)	T2 (600 *μ*g/L)	T3 (900 *μ*g/L)
ROS (optical density)				
10	0.56 ± 0.03	0.57 ± 0.01	0.63 ± 0.01	0.71 ± 0.02∗
20	0.53 ± 0.01	0.59 ± 0.02	0.65 ± 0.07∗	0.74 ± 0.03∗
30	0.57 ± 0.01	0.62 ± 0.02	0.70 ± 0.05∗	0.78 ± 0.07∗
TBARS (nmol/TBARS formed/mg protein/min)				
10	28.51 ± 1.51	30.21 ± 1.11	35.92 ± 0.5∗	39.63 ± 1.39∗
20	29.08 ± 1.63	31.08 ± 1.16	37.07 ± 0.6∗	41.06 ± 1.83∗
30	29.72 ± 1.71	33.79 ± 1.17	37.79 ± 0.7∗	41.83 ± 1.77∗
Reduced GSH (*μ*mol/g tissue)				
10	7.70 ± 0.3	6.45 ± 0.3	5.21 ± 0.2∗	3.95 ± 0.2∗
20	7.66 ± 0.3	6.35 ± 0.2	5.18 ± 0.2∗	3.82 ± 0.2∗
30	7.54 ± 0.3	6.31 ± 0.2	5.10 ± 0.2∗	3.79 ± 0.2∗
*Antioxidant enzymes*				
SOD (units/mg protein)				
10	15.51 ± 0.36	13.53 ± 0.35	11.56 ± 0.33∗	9.55 ± 0.32∗
20	15.40 ± 0.36	13.14 ± 0.35	10.99 ± 0.33∗	8.77 ± 0.32∗
30	15.26 ± 0.36	13.10 ± 0.35	10.86 ± 0.33∗	8.68 ± 0.32∗
CAT (units/min)				
10	5.12 ± 0.1	4.58 ± 0.09	3.84 ± 0.09∗	3.46 ± 0.07∗
20	5.08 ± 0.1	4.56 ± 0.09	3.78 ± 0.08∗	3.43 ± 0.07∗
30	5.04 ± 0.1	4.45 ± 0.09	3.62 ± 0.08∗	3.30 ± 0.06∗
POD (units/*μ*g)				
10	5.98 ± 0.13	5.33 ± 0.13	4.17 ± 0.11∗	4.04 ± 0.10∗
20	5.92 ± 0.13	5.30 ± 0.12	4.13 ± 0.11∗	3.95 ± 0.10∗
30	5.89 ± 0.13	5.27 ± 0.12	4.03 ± 0.10∗	3.89 ± 0.10∗

In each row, values (Mean ± SE) bearing asterisks differ significantly (*P* ≤ 0.05) from that of values in untreated (T0 negative control) fish. T1, T2, and T3 are positive control and dose based.

The article "Evaluation of DNA Damage, Biomarkers of Oxidative Stress, and Status of Antioxidant Enzymes in Freshwater Fish (Labeo rohita) Exposed to Pyriproxyfen" was published in 2022. Journal: Oxid Med Cell Longev.

**Table 4:** Oxidative stress parameters and antioxidant enzyme levels in *Labeo rohita* gills tissues subjected to pyriproxyfen dosages.

Parameters/days	Groups/treatment			
	T0 (0.0)	T1 (300 *μ*g/L)	T2 (600 *μ*g/L)	T3 (900 *μ*g/L)
ROS (optical density)				
10	0.34 ± 0.03	0.37 ± 0.01	0.49 ± 0.07∗	0.55 ± 0.09∗
20	0.35 ± 0.05	0.39 ± 0.04	0.53 ± 0.06∗	0.57 ± 0.07∗
30	0.37 ± 0.04	0.41 ± 0.01	0.56 ± 0.08∗	0.59 ± 0.09∗
TBARS (nmol/TBARS formed/mg protein/min)				
10	40.67 ± 1.63	44.47 ± 2.12	58.27 ± 2.22∗	61.07 ± 2.33∗
20	41.13 ± 2.61	44.88 ± 2.31	58.64 ± 3.41∗	62.39 ± 2.29∗
30	41.20 ± 1.61	45.04 ± 1.36	61.82 ± 2.39∗	63.70 ± 2.27∗
Reduced GSH (*μ*mol/g tissue)				
10	2.58 ± 0.05	2.24 ± 0.10	1.90 ± 0.04∗	1.56 ± 0.16∗
20	2.44 ± 0.11	2.23 ± 0.14	1.83 ± 0.03∗	1.52 ± 0.17∗
30	2.34 ± 0.15	2.05 ± 0.17	1.76 ± 0.08∗	1.47 ± 0.25∗
*Antioxidant enzymes*				
SOD (units/mg protein)				
10	10.79 ± 1.2	9.73 ± 1.12	8.98 ± 0.04	7.24 ± 0.12∗
20	10.68 ± 1.1	9.53 ± 1.17	8.13 ± 0.21∗	7.22 ± 0.18∗
30	10.57 ± 1.4	9.32 ± 1.11	8.07 ± 0.13∗	6.83 ± 0.31∗
CAT (units/min)				
10	3.03 ± 0.14	2.89 ± 0.12	2.48 ± 0.08	2.19 ± 0.13∗
20	2.98 ± 0.11	2.79 ± 0.17	2.33 ± 0.08∗	2.15 ± 0.19∗
30	2.95 ± 0.09	2.73 ± 0.15	2.19 ± 0.14∗	2.08 ± 0.21∗
POD (units/*μ*g)				
10	0.41 ± 0.05	0.37 ± 0.01	0.36 ± 0.01	0.26 ± 0.03∗
20	0.40 ± 0.04	0.36 ± 0.02	0.30 ± 0.05∗	0.24 ± 0.04∗
30	0.39 ± 0.05	0.34 ± 0.04	0.29 ± 0.06∗	0.22 ± 0.02∗

In each row, values (Mean ± SE) bearing asterisks differ significantly (*P* ≤ 0.05) from that of values in untreated (T0 negative control) fish. T1, T2, and T3 are positive control and dose based.

**Table 5:** Oxidative stress parameters and antioxidant enzyme levels in *Labeo rohita* brain tissue subjected to pyriproxyfen dosages.

Parameters/days	Groups/treatments			
	T0 (0.0)	T1 (300 *μ*g/L)	T2 (600 *μ*g/L)	T3 (900 *μ*g/L)
ROS (optical density)				
10	0.48 ± 0.02	0.50 ± 0.02	0.51 ± 0.03	0.53 ± 0.03
20	0.46 ± 0.02	0.52 ± 0.02	0.59 ± 0.03∗	0.72 ± 0.04∗
30	0.51 ± 0.02	0.53 ± 0.03	0.66 ± 0.03∗	0.76 ± 0.04∗
TBARS (nmol/TBARS formed/mg protein/min)				
10	18.60 ± 2.11	19.29 ± 1.03	20.97 ± 1.12	21.66 ± 1.06
20	19.08 ± 2.01	20.77 ± 1.21	26.46 ± 1.13∗	30.14 ± 1.13∗
30	19.18 ± 2.04	22.92 ± 1.5	26.66 ± 1.17∗	30.40 ± 2.13∗
Reduced GSH (*μ*mol/g tissue)				
10	3.01 ± 0.06	2.96 ± 0.06	2.79 ± 0.05	2.89 ± 0.04
20	2.96 ± 0.06	2.77 ± 0.05	2.66 ± 0.04	1.77 ± 0.03∗
30	2.88 ± 0.06	2.75 ± 0.05	2.10 ± 0.04∗	1.73 ± 0.03∗
*Antioxidant enzymes*				
SOD (units/mg protein)				
10	13.65 ± 0.3	12.09 ± 0.3	12.02 ± 0.2	11.96 ± 0.2
20	13.56 ± 0.3	12.20 ± 0.2	11.73 ± 0.2	8.87 ± 0.1∗
30	13.45 ± 0.3	11.88 ± 0.2	10.32 ± 0.2∗	8.75 ± 0.1∗
CAT (units/min)				
10	4.16 ± 0.08	3.93 ± 0.08	3.85 ± 0.07	3.76 ± 0.06
20	4.12 ± 0.08	3.68 ± 0.08	3.77 ± 0.07	2.46 ± 0.06∗
30	4.07 ± 0.08	3.59 ± 0.07	2.98 ± 0.07∗	2.23 ± 0.06∗
POD (units/*μ*g)				
10	3.04 ± 0.06	2.79 ± 0.06	2.64 ± 0.05	2.59 ± 0.04
20	3.01 ± 0.06	2.73 ± 0.05	2.35 ± 0.05	1.98 ± 0.04∗
30	3.03 ± 0.06	2.69 ± 0.05	2.03 ± 0.05∗	1.94 ± 0.04∗

In each row, values (Mean ± SE) bearing asterisks differ significantly (*P* ≤ 0.05) from that of values in untreated (T0 negative control) fish. T1, T2, and T3 are positive control and dose based.

The article "Evaluation of DNA Damage, Biomarkers of Oxidative Stress, and Status of Antioxidant Enzymes in Freshwater Fish (Labeo rohita) Exposed to Pyriproxyfen" was published in 2022. Journal: Oxid Med Cell Longev.

**Table 6:** DNA damage in different visceral organs of *Labeo rohita* (as observed by Comet assay) treated with various doses of pyriproxyfen.

Parameters/days	Groups/treatment			
	T0 (0.0)	T1 (300 *μ*g/L)	T2 (600 *μ*g/L)	T3 (900 *μ*g/L)
DNA damage by comet assay in liver				
10	2.35 ± 0.04	2.37 ± 0.05	2.39 ± 0.03	3.42 ± 0.14∗
20	2.37 ± 0.09	2.42 ± 0.06	3.47 ± 0.02∗	4.52 ± 0.19∗
30	2.43 ± 0.02	2.56 ± 0.02	4.70 ± 0.01∗	4.84 ± 0.22∗
DNA damage by comet assay in kidneys				
10	2.55 ± 0.19	2.67 ± 0.17	2.69 ± 0.27	4.47 ± 0.45∗
20	2.57 ± 0.21	2.72 ± 0.16	4.87 ± 0.51∗	5.53 ± 0.49∗
30	2.63 ± 0.25	2.76 ± 0.21	5.70 ± 0.61∗	5.81 ± 0.28∗
DNA damage by comet assay in gills				
10	2.23 ± 0.23	2.41 ± 0.11	2.51 ± 0.21	3.94 ± 0.44∗
20	2.31 ± 0.31	2.44 ± 0.14	3.87 ± 0.02∗	4.55 ± 0.39∗
30	2.23 ± 0.26	2.46 ± 0.12	4.77 ± 0.01∗	5.89 ± 0.42∗

In each row, values (Mean ± SE) bearing asterisks differ significantly (*P* ≤ 0.05) from that of values in untreated (T0 negative control) fish. T1, T2, and T3 are positive control and dose based.

## Data Availability

The data that support the findings of this study are available from the corresponding author upon reasonable request.

## Abbreviations

ANOVA: Analysis of variance
ATP: Adenosine triphosphate
CAT: Catalase
GSH: Glutathione
POD: Peroxidase
PPF: Pyriproxyfen
ROS: Reactive oxygen species
SOD: Superoxide dismutase
TBARS: Thiobarbituric acid reactive species.
